RETRACTED

# MicroRNA-219-2-3p Functions as a Tumor Suppressor in Gastric Cancer and Is Regulated by DNA Methylation

**DOI:** 10.1371/journal.pone.0060369

**Published:** 2013-04-23

**Authors:** Huizi Lei, Dongling Zou, Zheng Li, Min Luo, Lei Dong, Bin Wang, Haixin Yin, Yanni Ma, Changzheng Liu, Fang Wang, Junwu Zhang, Jia Yu, Yu Li

**Affiliations:** 1 Department of Pathology, Chongqing Medical University, Chongqing, People's Republic of China; 2 Department of Biochemistry, Institute of Basic Medical Sciences, Chinese Academy of Medical Sciences & Peking Union Medical College, Beijing, People's Republic of China; 3 Department of Gynecologic Oncology, Chongqing Cancer Institute, Chongqing, People's Republic of China; 4 Department of Orthopedic Surgery, Peking Union Medical College Hospital, Peking Union Medical College, Beijing, People's Republic of China; Wayne State University, United States of America

## Abstract

**Background & Aims:**

Gastric cancer is the most frequent gastrointestinal tumor in adults and is the most lethal form of human cancer. Despite of the improvements in treatments, the underlying mechanism of gastric carcinogenesis is not well known. To define novel modulators that regulate susceptibility to tumorgenesis, we focused on miR-219-2-3p.

**Methods:**

Quantitative RT-PCR was employed to investigate the level of miR-219-2-3p in gastric cancer (GC) tissues (n = 113) and their matched adjacent normal tissues (n = 113). In vitro cell proliferation, apoptosis assays, cell migration, and invasion assays were performed to elucidate biological effects of miR-219-2-3p. Since silencing of miRNA by promoter CpG island methylation may be an important mechanism in tumorgenesis, GC cells were treated with 5-aza-2′-deoxycytidine and trichostatin A, and expression changes of miR-219-2-3p were subsequently examined by quantitative RT-PCR. Finally, the methylation status of CpG island upstream of miR-219-2-3p was analyzed by methylation-specific PCR in GC tissues (n = 22).

**Results:**

miR-219-2-3p was down-regulated in GC and cell lines. In addition, the experiments documented the lower expression of miR-219-2-3p in GC specimens with higher grade and later stage tumors. Meanwhile, miR-219-2-3p exerted antiproliferative, proapoptotic, and antimetastatic roles and reduced levels of p-ERK1/2 in GC cells. Furthermore, 5-aza-2′-deoxycytidine and trichostatin A increased the expression (∼2 fold) of miR-219-2-3p in GC cells. By methylation-specific PCR, DNA methylation in the upstream region of miR-219-2-3p was detected in both adjacent normal tissues and cancer tissues. As expected, the methylation level was considerably higher in the miR-219-2-3p down-regulated group than up-regulated group.

RETRACTED

**Conclusions:**

miR-219-2-3p is potentially involved in gastric cancer progression and metastasis by regulating ERK1/2-related signal pathways, which may provide a novel therapeutic strategy for treatment of gastric cancer. Methylation mechanism may be involved in modulating the expression level of miR-219-2-3p in gastric cancer.

## Introduction

Gastric cancer (GC) is the 4^th^ most common cancer and the second-highest cause of cancer death worldwide. Nowadays, patients with late-stage GC are with an overall 5-year survival of approximately 20%[1]. Cancer develops as a result of an accumulation of various endogenous and exogenous causes. Eating habits and a increase in Helicobacter pyloriinfection are important exogenous causes for GC[2], while genetic, as well as dietary, levels of the hormone gastrin[3], and other chronic gastric inflammation-causing factors are found to be associated with predisposition to cancer development. Gene alterations play an important role in GC, and alterations in a large number of oncogenes and tumor suppressor genes have already been reported in GC.

Some prognostic tumor biomarkers in GC such as human epidermal growth factor receptor 2 (HER2), vascular endothelial growth factor (VEGF), epidermal growth factor receptor (EGFR), have been associated with disease characteristics and can therefore be used to inform patient management. For example, patients with tumors that test positive for HER2 can be treated with trastuzumab plus chemotherapy[4], and patients with tumors that test positive for VEGF can be treated with bevacizumab plus chemotherapy[5]. However, the molecular mechanisms underlying the development of GC remain a challenge, thus additionally informative biomarkers are urgently needed.

MicroRNAs (miRNA) are a class of small RNA molecules involved in regulation of translation and degradation of mRNAs[6]. MiRNAs bind to complementary sequences in the 3′ untranslated regions (UTR) of their target mRNAs and induce mRNA degradation or translational repression[7]. Most known functions of miRNAs are related to negative gene regulation: miRNAs silence gene expression, usually by interfering with mRNA stability or protein translation. In recent years, miRNAs were believed to act as oncogene or tumor suppressor gene, and contribute to cancer initiation and progression by regulating gene expression[8]. The discovery of cancer-specific upstream region hypermethylation of numerous miRNAs has demonstrated an epigenetic mechanism for aberrant miRNA expression[9], [10].

In human and mice, there are two genomic loci (miR-219-1 and miR-219-2) which encode miR-219 precursor transcripts. miR-219-1 is located on chromosome 6 (MI0000296) and mir-219-2 is located on chromosome 9 (MI0000740)[11] (**Fig. 1A**). Processing of the precursor transcripts by dicer generates three mature miRNAs: miR-219-5p from the 5′ ends of both precursors, and miR-219-1-3p and miR-219-2-3p from the 3′ end of pre-miR-219-1 and pre-miR-219-2, respectively. Since the seed region of these three mature products is unique, each miRNA is predicted to regulate unique targets. Although miR-219-5p is known to be down-regulated in multiple cancer such as malignant astrocytoma[12] and hepatocellular carcinoma[13], the expression of miR-219-1-3p and miR-219-2-3p has not been studied. Interestingly, miR-199b and miR-219-2-3p genes are located at proximity to a segment of chromosome 9q34.11 (**Fig. 1A**). A previous study shown that miR-199b-5p was down-regulated in medulloblastoma by methylation of a CpG island 3 kb upstream of the 5′-site of miR-199b-5p promoter[14]. Since DNA methylation can affect large regions of chromatin and regulate the transcription of distant genes, it is necessary to investigate whether miR-219-2-3p is down-regulated and regulated by methylation as miR-199b-5p in cancer. In this study, we found that miR-219-2-3p was down-regulated in GC tissues and associated with progressive phenotypes of GC. Moreover, re-introduction of miR-219-2-3p reduced the viability of GC cells and induced cell apoptosis, suggesting that miR-219-2-3p was a candidate tumor suppressor in GC. Further methylation analysis of miR-219-2-3p promoter indicated that its expression was regulated by methylation of correlated CpG islands to some extent. Finally, we found that miR-219-2-3p acted as a tumor suppressor through inhibiting the activity of ERK1/2 signal pathway in GC cells.

RETRACTED

**Figure 1:** The expression of miR-219-2-3p in gastric cancer tissues and cell lines. (A) Schematic showing human mir-219-1 and mir-219-2 genomic structures. Processing of the precursor transcripts generates the same miR-219-5p and two unique miRNAs, 219-1-3p and 219-2-3p. (B) MiR-219-2-3p was detected in 113 GC patients by real-time -PCR. Data is presented as log 2 of fold change of GC tissues relative to non-tumor adjacent tissues. (C) Expression levels (as log 2 of fold change of GC tissues relative to non-tumor adjacent tissues) of miR-219-2-3p in I–II stages (n = 39) versus III–IV stages (n = 71) of the cancer patients. (D) The four patients who were diagnosed as gastric cancer in H&E staining (original magnification, x100). (E) Expression levels of miR-219-2-3p were examined by real-time PCR in four patients as described in fig.1D and four GC cell lines. Experiments were performed three times. All data uses independent t test and is shown as mean ± SD. *, *P*<0.05.

RETRACTED

## Results

### miR-219-2-3p was differentially expressed in GC and GC cell lines

To assess the expression of miR-219-2-3p in GC, TaqMan RT-PCR analysis was conducted in 113 pairs of GC tissues and matched adjacent normal tissue samples. As compared with normal tissue samples, more than half of the primary tumors exhibited low levels of miR-219-2-3p (58%, 65 of 113; **Fig. 1B**). Furthermore, four patients whose expression of miR-219-2-3p were significant down-regulated were chosen (**Fig. 1D**). The miR-219-2-3p expression in those patients and four GC cell lines (MGC-803, HGC-27, MKN-45, SGC-7901) was analyzed to reveal that miR-219-2-3p was also down-regulated in GC cells (**Fig. 1E**). These results suggested that down-regulated miR-219-2-3p was a frequent event in human GC and might be involved in gastric carcinogenesis. Because of the universal down-regulation of miR-219-2-3p in tested GC cell lines, MGC-803 and HGC-27 were randomly chosen for further study.

### Relationship between clinicopathological factors and miR-219-2-3p expression in GC

This study included 113 GC patients. To evaluate the correlation between miR-219-2-3p expression and clinicopathological characteristics, patients were divided into groups with down-regulation and up-regulation. As shown in **table 1** and **fig.1C**, a statistically significant association was observed between the expression of miR-219-2-3p and GC clinical stage. The patients with lower levels of miR-219-2-3p expression seemed to be associated with high-grade and late-stage tumors (p = 0.047, independent-samples t test). These data suggested that alterations of miR-219-2-3p could be involved in GC progression.

**Table 1:** Clinicopathologic characteristics of patients with GC.

Parameter	Total	Percentage	95%CI of mean log2 fold		P
	samples		change±SEM		
Age(years)					
≥60	112	47.3%	−0.307	(−0.969–0.355)	0.847
<60		52.7%	−0.216	(−0.877–0.444)	
Gender					
Male	112	84.8%	−0.413	(−0.918–0.091)	0.118
Female		15.2%	0.601	(−0.561–1.762)	
Location					
Proximal	113	30.9%	−0.124	(−0.956–0.708)	0.765
Body		41.6%	−0.45	(−1.125–0.225)	
Distal		27.4%	−0.085	(−1.097–0.927)	
Lauren's classification					
Intestinal	72	18.1%	0.765	(−0.999–2.528)	0.397
Diffuse		68.1%	−0.213	(−0.912–0.485)	
Mixed		13.9%	−0.508	(−2.283–1.268)	
Grade					
Well and Moderate	62	21.0%	0.434	(−1.324–2.192)	0.366
differentiated					
Poorly differentiated		79.0%	−0.297	(−1.010–0.416)	
Tumor size					
T1–T2	111	17.1%	0.282	(−0.701–1.264)	0.286
T3		21.6%	0.174	(−0.985–1.334)	
T4		61.3%	−0.539	(−1.136–0.058)	
Lymphatic invasion					
N0–N1	111	67.6%	−0.143	(2.436–0.281)	0.533
N2–N3		32.4%	−0.457	(−1.323–0.410)	
Nodal involvement					
Negative	110	90.9%	−0.314	(−0.806–0.178)	0.306
Positive		9.1%	−0.008	(−1.526–1.510)	
Stage					
I–II	110	35.5%	0.387	(−0.420–1.195)	0.047^*^
III–IV		64.5%	−0.591	(−1.165–0.018)	
Perineural Invasion					
Negative	81	56.8%	−0.174	(−0.838–0.490)	0.634
Positive		43.2%	−0.424	(−1.265–0.417)	
Ki67					
1+2	27	25.9%	0.925	(−2.863–4.713)	0.163
3+4		74.1%	−0.724	(−1.789–0.341)	
Her2 amplification					
Negative	41	48.8%	−0.227	(−1.309–0.855)	0.348
Positive		51.2%	0.039	(−1.044–1.121)	
Top2a					
0+1	42	42.9%	−0.0988	(−1.120–0.923)	0.957
2+3		57.1%	0.134	(−1.014–1.283)	
CA199					
<37	29	75.9%	0.092	(−0.859–1.042)	0.258
>37		24.1%	−1.115	(−4.032–1.802)	
CA724					
<6.1	28	67.9%	−0.424	(−1.226–0.378)	0.538
>6.1		32.1%	0.135	(−2.724–2.994)	

RETRACTED

### Overexpression of miR-219-2-3p in GC cells inhibits cell proliferation and cell survival

The remarkable reduction of miR-219-2-3p expression in GC samples promoted us to explore the possible biological significance of miR-219-2-3p in tumorgenesis. Given that miR-219-2-3p played a role in the regulation of cell proliferation[15], MGC-803 and HGC-27 cells were transfected with miR-219-2-3p and scramble mimics and analyzed for cell growth, cell apoptosis and cell cycle progression respectively. First of all, RT-PCR was used to measure the level of miR-219-2-3p after overexpression experiments. We found that miR-219-2-3p increased by more than 100 folds in miRNA transfected MGC-803 and HGC-27 cells (**Fig.2A**). Furthermore, the CCK-8 proliferation assay shown that cell growth rate was reduced in miR-219-2-3p mimics-transfected MGC-803 and HGC-27 cells when compared with scramble-transfected cells or untreated cells (**Fig. 2B**). After transfection, the inhibition ratio was 26% (48 h) and 28% (96 h) in the MGC-803 cells and 13% (72 h) and 14% (96 h) in HGC-27 cells. These results suggested that miR-219-2-3p was indeed involved in the negative regulation of cell growth. However, there was no significant effect on cell cycle arrest in miR-219-2-3p treated GC cells (**Fig. S1**). To address whether up-regulation of miR-219-2-3p would induce GC cell apoptosis and cell death, the number of early apoptotic MGC-803 and HGC-27 cells following treatment with miR-219-2-3p mimics was examined. As expected, few early apoptotic cells (10% in MGC-803 or 2.9% in HGC-27) were detected in the scramble-treated cells, whereas miR-219-2-3p mimics treatment increased the percentage of early apoptotic cells (17.5% in MGC-803 or 8.3 in HGC-27) as judged by Annexin V staining (**Fig. 2C**). Therefore, we concluded that miR-219-2-3p could affect cell survival in GC cells.

**Figure 2:** Overexpression of miR-219-2-3p inhibits gastric cancer cell growth and affects cell apoptosis. (A) Expression levels of miR-219-2-3p were examined by real-time PCR after transfection with 50 nmol/L of miR-219-2-3p mimics or scramble or no transfection. (B) Growth of MGC-803 and HGC-27 cells was shown after transfection with 50 nmol/L of miR-219-2-3p mimics or scramble or no transfection. The growth index was assessed at 1, 2, 3, 4, and 5 d. (C) MGC-803 and HGC-27 cells were stained with PE Annexin V and 7-AAD 72 h after treatment with miR-219-2-3p mimics or scramble. Early apoptotic cells are shown in the right quadrant. *, *P*<0.05; ***, *P*<0.001.

RETRACTED

### Overexpression of miR-219-2-3p in GC cells inhibits cell migration and invasion

To further detect whether miR-219-2-3p is associated with progression of GC, wound healing and transwell assay were performed to analyze the effect of miR-219-2-3p expression on the migratory and invasive behavior of MGC-803 and HGC-27 cells. We found that introduction of miR-219-2-3p into MGC-803 and HGC-27 cells resulted in a significant reduction of cell migration during the closing of an artificial wound created over a confluent monolayer (**Fig. 3A**). These cells were maintained in serum-free medium during the course of wound healing to ensure that any augmented migratory behavior could not be affected by altered cell proliferation. In addition, restoration of miR-219-2-3p dramatically inhibited the normally strong invasive capacity of MGC-803 and HGC-27 cells, which carried low endogenous level of miR-219-2-3p (**Fig. 3B**). These results indicated that miR-219-2-3p overexpression contributes to regulation of GC cell motility and progression in vitro.

**Figure 3:** Overexpression of miR-219-2-3p inhibits gastric cancer cell migration and invasion. (A) MGC-803 and HGC-27 cells were not transfected or transfected with 50 nmol/L of miR-219-2-3p mimics or scramble for 24 hours, and wounds were made. The relative ratio of wound closure per field is shown. (B) MGC-803 and HGC-27 cells were not transfected or transfected with 50 nmol/L of miR-219-2-3p mimics or scramble for 24 hours, and transwell invasion assay was performed. The relative ratio of invasive cells per field is shown. Magnification for identification of migration is ×400 and invasion is ×40. All data is shown as mean ± SD.

### MiR-219-2-3p expression is epigenetically regulated

Based on the above findings, we conclude that miR-219-2-3p was an important regulator in GC. However, the regulatory mechanisms of miR-219-2-3p expression were still unknown. Since many miRNAs were identified as targets of methylation regulation, such as miR-9, miR-34b/c and miR-148a in metastatic carcinomas[16], and miR-137 and miR-193a in oral cancer[17], miR-193b and miR-145 in prostate cancer[18], [19], we decided to analyze the regulatory mechanism of miR-219-2-3p expression from its genomic methylation. After analyzing the genomic region spanning the miR-219-2-3p gene, we identified a large CpG island (**Fig. 4A**). To investigate whether miR-219-2-3p was epigenetically regulated in GC, MGC-803, HGC-27 cells were treated with demethyltransferase inhibitor, 5-aza-2′-deoxycytidine (5-Aza-CdR) and the histone-deacetylase inhibitor trichostatin A (TSA). Then the expression of miR-219-2-3p by RT-PCR was analyzed (**Fig. 4B**). The results shown that the expression of miR-219-2-3p was up-regulated in two situations: for the 5-Aza-CdR treatment, the expression of miR-219-2-3p was up-regulated in MGC-803 (5-Aza-CdR 1.5 µmol/L; 2.14-fold) and HGC-27 (5-Aza-CdR 0.5 µmol/L; 3.07-fold) compared with DMSO treated control group; for the 5-Aza-CdR and TSA combination treatment, the expression of miR-219-2-3p was much higher in MGC-803 (5-Aza-CdR 1.5 µmol/L; 1.98-fold) and HGC-27 (5-Aza-CdR 1.5 µmol/L; 1.28-fold) compared with TSA control group. These results indicated that epigenetic factors could affect miR-219-2-3p expression in GC. Synergy of demethylation and histone deacetylase inhibition led to the re-expression of miR-219-2-3p in GC. To further detect whether miR-219-2-3p was associated with methylation of GC, we examined the methylation status of the miR-219-2-3p upstream region using methylation-specific PCR (MSP; **Fig. 4C**). 22 pairs of tissues (primary tumors and their matched adjacent normal tissues) in the 113 pairs were chosen, including 11 patients who possessed lower miR-219-2-3p levels (down-regulation group) and 11 patients who possessed higher miR-219-2-3p levels (up-regulation group). We found that DNA methylation in upstream regions of miR-219-2-3p existed in both adjacent normal tissues and cancer tissues. However, the hypermethylation ratio of upstream region of miR-219-2-3p gene in the down-regulation group was 63.6% (7 of the 11), which was higher than the up-regulation group (36.3%, 4 of the 11). These results suggested that the methylation level of the upstream CpG region of miR-219-2-3p was higher in the miR-219-2-3p down-regulated group than in the up-regulated one.

RETRACTED

**Figure 4:** Down-regulation of miR-219-2-3p in gastric cancer cells is associated with methylation of miR-219-2-3p upstream region. (A) A schematic illustration of deletion of a segment (90 M–141 M) of chromosome 9q34.11 where the miR-219-2-3p genes located. (B) Effect of 5-Aza-CdR and TSA on miR-219-2-3p expression in MGC-803 and HGC-27 gastric cancer cell lines. 5-Aza-CdR or 5-Aza-CdR combination with TSA significantly increased miR-219-2-3p levels. (C) Representative MSP results of miR-219-2-3p methylation in primary gastric cancer tumors and normal adjacent tumor tissues. Case numbers are shown on top. M: methylated primers; U: unmethylated primers. Cases with hypermethylation were marked.

### Overexpression of miR-219-2-3p dampens ERK1/2 signaling pathway

Activation of ERK1/2 pathway was well documented in various tumor types, such as GC[20], pancreatic cancer[21] and breast cancer[22]. Previous studies have shown the importance of ERK1/2 signaling pathway in the regulation of migration, invasion and metastasis of cancer cell lines[23]. To investigate whether miR-219-2-3p affects cell activities through ERK1/2 pathway, the phosphorylation level of ERK1/2 in MGC-803 and HGC-27 cells was examined after miR-219-2-3p overexpression. Cellular levels of p-ERK1/2 significantly decreased in miR-219-2-3p mimics–transfected cells as compared with scramble-transfected or untreated cells. However, no obvious difference was observed in total ERK1/2 level (**Fig. 5A**). These findings suggested that the accelerated GC cell growth might be partially due to activated ERK1/2 pathways.

**Figure 5:** miR-219-2-3p inhibits activation of p-ERK1/2. (A) MGC-803 and HGC-27 cells untreated and transfected with scrambled or miR-219-2-3p mimics were subjected to western blot analysis of phosphorylated ERK1/2, total ERK1/2 and GAPDH (as a loading control). The data shown is representative of three individual western blot analyses. (B) The candidate onco-targets of miR-219-2-3p forecast by TargetScan Release 5.2, and miRDB. (C) Bioinformatically and functionally implicated miR-219-2-3p in GC.

### Bioinformatics approach to search for potential targets of miR-219-2-3p

MiRNAs modulate gene expression by interacting with their target mRNAs resulting in mRNA degradation or translational repression. To further investigate the mechanism of miR-219-2-3p in GC, we bioinformatically (TargetScan Release 5.2 and miRDB) and functionally implicated miR-219-2-3p in GC, and found the genes targeted by miR-219-2-3p (**Table S2**). Among the 371 predicted targets of miR-219-2-3p, 31 of them shown high potential since they were predicted by both programs, while others were only predicted by one of the programs. Of these 31 genes, ERBB3, MAPK8, SCL7A11, YOD1, TBK1, SOX4 were found to be oncogene or apoptosis-related genes by previous published papers. (**Fig. 5B and 5C**).

## Discussion

In recent years, accumulated evidence has led oncologists to speculate that unrevealed molecular factors, particularly non-coding RNAs previously classified as “junk,” play important roles in tumorigenesis and tumor progression. Depending on their mRNA targets, miRNAs can function as tumor suppressors or promoters of oncogenesis. However, the mechanisms that dysregulated miRNAs have not been widely studied, including aberrant miRNA biogenesis and transcription[24], [25], epigenetic alteration[26], [27], and amplification or loss of genomic regions that encode miRNAs[28].

RETRACTED

As shown in this report, we analyzed the expression of miR-219-2-3p in 113 GC patients and found that the levels seem to be lower in GC. Although miR-219-2-3p has been reported to be closely related to diabetic retinopathy[29], oligodendrocytes[15], alzheimer disease [30]and glioblastoma[12], its function in GC remains to be determined. Furthermore, we shown that re-expression of miR-219-2-3p in GC cells resulted in the induction of cell apoptosis and reduced cell viability. These results allowed us to speculate that down-regulation of miR-219-2-3p might provide a survival advantage to GC cells. However, the mechanism responsible for miR-219-2-3p down-regulation in GC is still unknown. Because the loss at 9q34.11, where miR-219-2-3p is located, is rarely detected in GC [31], it is unlikely that allelic loss is responsible for its down-regulation. On the other hand, we found that miR-219-2-3p was markedly up-regulated when GC cells, MGC-803 and HGC-27, were treated with both 5-Aza-CdR and TSA. In addition, computational analysis reveals that miR-219-2-3p is located in a CpG island on chromosome 9q34.11. Therefore, it seems possible that DNA methylation and histone deacetylation may be associated with miR-219-2-3p regulation. By MSP, samples methylation frequencies detected in the upstream region of miR-219-2-3p was higher in the miR-219-2-3p down-regulated group than in the up-regulated group. This specificity furnished the hypothesis of a relationship between miR-219-2-3p expression and DNA methylation. Overall, the results suggested that methylation was an important mechanism for miR-219-2-3p down-regulation in GC.

We performed prediction by TargetScan and miRDB programs and found that 6 genes could be potential targets of miR-219-2-3p. Among the candidate targets of miR-219-2-3p, the receptor tyrosine kinases ERBB3 (epidermal growth factor receptor family) drew our attention. High levels of ERBB3 is strongly associated with tumor progression and poor prognosis of patients with GC[32]-[34] and the EGFR kinase inhibitors gefitinib could prevent EGFR and ERBB2 activation of ERBB3. Meanwhile, ERBB3 expression also serves as an effective predictor of sensitivity to gefitinib[35]. It is known that repressed ERBB3 transcription inhibits signaling cascades from ERK1/2 pathways[36]. However, the predicted target genes need to be further experimentally validated. Moreover, miRNAs may function according to a combinatorial circuits model, in which a single miRNA may target multiple mRNAs, and several coexpressed miRNAs may target a single mRNA. Recent studies have suggested that the biological concept of ‘one hit–multiple targets’ could be used in clinical therapeutics[37]. It is likely that a specific miRNA may function through cooperative down-regulation of multiple targets and miRNAs function also by suppressing the translation of their target genes. To explore the full impact of a miRNA, genome-wide proteomic studies should be done.

RETRACTED

In conclusion, our expression and functional studies suggested that miR-219-2-3p was differentially expressed by methylation mechanism and had a tumoral suppression function by regulating ERK1/2-related signal pathways in GC. Meanwhile, the lower expression of miR-219-2-3p in GC specimens was correlated with higher grade and later stage. Reintroducing expression of miR-219-2-3p on GC cells suppressed cell proliferation, migration, invasion and induced apoptosis indicated that miRNA-based theraputic pattern might serve as a basis for the development of novel potential therapies in gastric cancer.

## Materials and Methods

### Tissue Specimens

Gastric tumors and their morphologically normal tissues (located >3 cm away from the tumor) were obtained between November 2009 and November 2011 from 113 GC patients undergoing surgery at Cancer Hospital of Chinese Academy of Medical Sciences(CICAMS, n = 21), Chinese PLA General Hospital (301 hospital, n = 31), and The First Affiliated Hospital of Shanxi Medical University (n = 61). The use of the tissue samples for all experiments was approved by the ethical board of the Institute of Basic Medical Sciences, Chinese Academy of Medical Sciences. All participants provided their verbal informed consent to participate in this study, and their verbal informed consents were written down. This consent process was also approved by the ethics board. Tissue samples were cut into two parts, one was fixed with 10% formalin for histopathological diagnosis, and the other was immediately snap-frozen in liquid nitrogen, and stored at −196°C in liquid nitrogen until RNA extraction. This group consisted of 95 males, 17 females and one without gender information with a median age of 58 years (range, 31–82 years).Formalin-fixed paraffin-embedded tissue blocks of GC were collected from the Cancer Hospital of Chinese Academy of Medical Sciences (CICAMS, n = 4) between 2009 and 2011. Due to individual differences between patients, we lacked information of some clinicopathologic data. The use of the tissue samples for all experiments was approved by all the patients and by Ethics Committee of the institution. The characteristics of patients are described in **Table 1**.

RETRACTED

### Cell Cultures and Transfection

A total of 4 human GC cell lines MGC-803 (mucinous gastric cancer, poorly differentiated), HGC-27 (metastatic lymph node, undifferentiated carcinoma), MKN-45 (Signet ring carcinoma poorly differentiated), SGC-7901 (adenocarcinoma, moderately differentiated) were examined in this study. The MGC-803 HGC-27, MKN-45, SGC-7901 cell line was purchased from the Cell Resource Center of Institute of Basic Medical Sciences, Chinese Academy of Medical Sciences and Peking Union Medical College (Beijing, China). MGC-803 was propagated in Dulbecco's modified Eagle medium (Gibco; Invitrogen; Life Technologies, Germany), supplemented with 10% fetal bovine serum (FBS; PAA, Pasching, Austria) and streptomycin (100 µg/ml), penicillin (100 U/ml). The HGC-27, MKN-45, SGC-7901 were maintained in RPMI 1640 medium (PAA) supplemented with 10% FBS (PAA). The human GC cell lines MGC-803, HGC-27 were transfected with miR-219-2-3p mimics and negative control miRNA mimics (GenePharma; Shanghai, China, **Table S1**) at a final concentration of 10 nmol/L using Dharmafect 1(Thermo Fisher; IL, USA) in accordance with the manufacturer's instructions.

### TaqMan RT-PCR for miRNA Expression

Total RNA was extracted from the cells and tissues with Trizol reagent (Invitrogen, Calsbad, CA, USA). MiRNAs were quantitated by real-time PCR using TaqMan MicroRNA assay (Invitrogen, USA). First-strand complementary DNA (cDNA) synthesis was carried out from 1 µg of total RNA in 12 µl of final volume containing 2 M stem-loop primer, 10 mM dNTP Mix (Invitrogen, USA). The mix was plate at 65°C for 5 min, and then mixed with 5×RT buffer, 0.1 M DTT, 200 U/µl MultiScribe reverse transcriptase and 40 U/µl RNase inhibitor (Invitrogen, USA). The mix was plate at 37°C for 55 min, 70°C for 15 min and then held at −20°C. Real-time PCR was performed using a standard TaqMan PCR protocol. The 20 µl PCRs reactions included 1 µl of RT product, 1× Universal TaqMan Master Mix and 1× TaqMan probe/primer mix (Invitrogen, USA, **Table S1**). All RT reactions including no-template controls were run in triplicate. All mRNA quantification data was normalized to U6. The relative amount of transcript was calculated using the comparative Ct method.

### 5-Aza-CdR and Trichostatin A treatment of cell lines

GC cell lines MGC-803 were treated with 5-aza-2′-deoxycytidine(5-Aza-CdR;Sigma-Aldrich, USA) at 0.7 µmol/L,1.5 µmol/L,3 µmol/L and HGC-27 were treated with 5-Aza-CdR at 0.5 µmol/L,1 µmol/L,1.5 µmol/L for 3 days or 300 nmol/L trichostatin A (TSA; Sigma-Aldrich, USA) for 24 hours. For the combination treatment, cells were treated with 5-Aza-CdR for 48 hours firstly. Then TSA (300 nmol/L) was added, and the cells were treated for an additional 24 hours. Culture medium containing drug was replaced every 24 hours. RNA of cell lines was purified with TRIzol reagent following the instructions from the manufacturer. cDNA synthesis was carried out as described earlier, and 1 ml of the diluted cDNA for each sample was amplified by RT-PCR using the protocol previously described.

RETRACTED

### DNA isolation and bisulfite modification

Genomic DNA was obtained from −196°C in liquid nitrogen primary tumors, and their matched adjacent normal tissues (n = 22, include 11 patients which expression of miR-219-2-3p were down-regulated and the others were up-regulated) and used Biomed DNA Kit (Biomed, Beijing, China) according to the manufacturer instructions. Bisulfite treatment and recovery of samples were carried out with the Epitect Bisulfite kit (Qiagen; Hilden,Germany). Genomic DNA (2 µg) in 20 µl water was used for each reaction and mixed with 85 µl bisulfite mix and 35 µl DNA protect buffer. Bisulfite conversion was performed on a thermocycler as follows: 99°C for 5 min, 60°C for 25 min, 99°C for 5 min, 60°C for 85 min, 99°C for 5 min, 60°C for 175 min and 20°C indefinitely. The bisulfite-treated DNA was recovered by Epitect spin column and subsequently sequenced to confirm the efficiency of bisulfite conversion.

### Methylation analysis

MSP was used to analyze methylation of miR-219-2-3p upstream region in cell lines and tissues. Methprimer was used to design MSP primer (**Table S1**). MSP reactions on new primers were optimized using Methylated positive control (M-DNA), which using normal human peripheral lymphocyte DNA treated in vitro with Sss I methyltransferase (New England Biolabs, Beverly, MA). The DNA of two normal human peripheral lymphocytes was used as normal control. Touchdown PCR consisted of two phases: phase 1 included an initial denaturation of 95°C for 5 min, followed by 45 cycles of denaturation at 95°C for 30 s, annealing at variable temperatures for 30 s, and extension at 72°C for 40 s. In the first cycle, the annealing temperature was set to 58°C and, at each of the 10 subsequent cycles, the annealing temperature was decreased by 0.6°C. Phase 2 consisted of 35 cycles of 95°C for 30 s, 52°C for 30 s, and 72°C for 40 s. MSP products were analyzed on 3% polyacrylamide gels.

### Cell proliferation, apoptosis, and cell cycle assay

Cells were incubated in 10% CCK-8 (Dojindo; Kumamoto, Japan) diluted in normal culture medium at 37°C until visual color conversion occurred. Proliferation rates were determined at 0, 24, 48, 72, 96 hours after transfection. The absorbance of each well was measured with a microplate reader set at 450 nM and 630 nM. All experiments were performed in quadruplicate. The apoptosis assay was performed on MGC-803 and HGC-27 cell lines 72 hours after transfection using the PE Annexin V Apoptosis Detection Kit I (BD Pharmingen; San Diego, CA, USA) and analyzed by fluorescence-activated cell sorting (FACS). Cell cycle analysis was performed on MGC-803 and HGC-27 cell lines 48 hours after transfection with miR-219-2-3p mimics and scramble respectively. Cells were harvested, washed twice with cold PBS, fixed in ice-cold 70% ethanol, and incubated with propidium iodide (PI) and RNase A, then analyzed by FACS. Each sample was run in triplicate.

RETRACTED

### Cell migration and invasion assays

MGC-803 and HGC-27 cells were grown to confluence on 12-well plastic dishes and treated with scramble or miR-219-2-3p mimics. 24 hours after transfection, linear scratch wounds (in triplicate) were created on the confluent cell monolayers using a 200 µl pipette tip. To remove cells from the cell cycle prior to wounding, cells were maintained in serum-free medium. To visualize migrated cells and wound healing, images were taken at 0, 12, 24, 36, 48, 60 and 72 h hours. A total of ten areas were selected randomly from each well and the cells in three wells of each group were quantified. For the invasion assays, after 24 hours transfection, 1×10^5^ cells in serum-free media were seeded onto the transwell migration chambers (8 µm pore size; Millipore, Switzerland) which were coated with Matrigel(Sigma-Aldrich; St Louis, MO, USA) on the upper chamber. Media containing 20% FBS was added to the lower chamber. After 24 hours, the non-invading cells were removed with cotton wool, invasive cells located on the lower surface of the chamber were stained with May-Grunwald-Giemsa stain (Sigma Diagnostics; St Louis, Missouri, USA) and counted using a microscope (Olympus; Tokyo, Japan). Experiments were independently repeated three times.

### Protein isolation and western blotting

At the indicated times, MGC-803 cells and HGC-27 cells were harvested in ice-cold PBS and lysed on ice in cold preparation of modified radioimmunoprecipitation buffer supplemented with protease inhibitors. Protein concentration was determined by the BCA Protein Assay Kit (Bio-Rad, Milan, Italy) and equal amounts of proteins were analyzed by SDS–PAGE (10% acrylamide). Gels were electroblotted onto nitrocellulose membranes (Millipore, Bedford, MA, USA). For immunoblot experiments, membranes were blocked for 2 h with 5% non-fat dry milk in Tris-buffered saline containing 0.1% Tween-20, and incubated at 4°C over night with primary antibody. Detection was performed by peroxidase-conjugated secondary antibodies using the enhanced chemiluminescence system. Primary antibodies used were: GAPDH from Zhong-Shan JinQiao(Beijing, China); ERK1/2 (rabbit anti–ERK1/2, New England Biolab, NEB) and phospho-ERK1/2 (rabbit anti-phospho-ERK1/2, New England Biolab, NEB)

RETRACTED

### Histology

Tissues were fixed overnight in buffered formalin, embedded in paraffin, cut to 3-µm thickness, and stained with hematoxylin-eosin (H&E) staining.

### Bioinformatics and Statistical analyses of data

The miRNA targets predicted by computer-aided algorithms were obtained from miRDB (http://mirdb.org/miRDB/), targetscan5.2 (http://www.targetscan.org) and Statistical analysis were performed using SPSS 15.0. Data was presented as the mean ± standard deviation. Statistical analyses were done by analysis of variance (ANOVA) or Student's t test and statistical significance level was set at α = 0.05 (two-side).

## Supporting Information

Figure S1 **Overexpression of miR-219-2-3p has no significant effect on cell cycle in gastric cancer.**
(TIF)

Table S1 **Primer/mimics/probe sequence.**
(TIF)

Table S2 **Potential targets of miR-219-2-3p.**
(TIF)
